# Chelerythrine Chloride Inhibits Stemness of Melanoma Cancer Stem-Like Cells (CSCs) Potentially via Inducing Reactive Oxygen Species and Causing Mitochondria Dysfunction

**DOI:** 10.1155/2022/4000733

**Published:** 2022-06-18

**Authors:** Hong Li, Mei He, Pengyu Zhao, Ping Liu, Wei Chen, Xuewen Xu

**Affiliations:** ^1^Medical Cosmetology Department of Chengdu Second People's Hospital, Chengdu 610041, China; ^2^Aesthetic and Plastic Burn Surgery Department of West China Hospital, Sichuan University, Chengdu 610041, China

## Abstract

Growing evidence has demonstrated that high heterogeneity contributes to poor prognosis and malignancies. The existence of melanoma cancer stem-like cells (CSCs), which are a small subpopulation of melanoma cells, is responsible for tumour resistance to therapies. Recently, plant secondary metabolites have attracted attention because they are considered promising compounds that are isolated from herbs that could help to target different subpopulations of tumours. In the present study, we aimed to identify the antitumourigenic activities of the medicinal compound chelerythrine chloride (CHE) on melanoma CSCs. CHE (30-40 *μ*mol/L) induced apoptosis in A375 and A2058 CSCs. A relatively low dose of CHE (1-5 *μ*mol/L) inhibited the stemness of melanoma CSCs without inducing apoptosis. Coculture of CHE with A375 and A2058 cells also inhibited sphere formation and decreased stemness factors, including Nanog, Oct4, and Sox2. In functional characterizations, we observed that CHE treatment increased both cellular reactive oxygen species (ROS) and mitochondrial ROS, which resulted in a decrease in mitochondrial energy production and sphere formation. Abolishing CHE-induced ROS by N-acetyl-L-cysteine (NAC), a ROS scavenger, reversed the inhibitory effects of CHE on sphere formation, suggesting that CHE-induced ROS are the potential cause of the inhibition of sphere formation. In conclusion, CHE may exert its antitumour effect as an antistem cell natural compound, suggesting that selection of the antistem cell effects of natural compounds might be a promising strategy to overcome the poor prognosis of melanoma due to the presence of CSCs.

## 1. Introduction

Malignant melanoma (MM) is a highly aggressive form of skin cancer that continues to increase rapidly worldwide. Intratumoural heterogeneity is believed to be one of the key reasons for this aggressiveness in malignant melanoma. In fact, tumour cells are organized and maintained in layers by subpopulations of cells termed cancer stem cells (CSCs or tumour initiating cells). These cells have stem cell-like functional properties, such as self-renewal and multipotency [1, 2]. The existence of CSCs is believed to contribute to tumour initiation, maintenance, progression, metastasis, and recurrence. Moreover, because of their unique biological characteristics, CSCs remarkably result in an increase in radioresistance and chemoresistance, which leads to poor prognosis. In addition, the CSC phenotype of the tumour is not a strict state, and the intratumoural heterogeneity of the tumour extends to CSC features, mainly due to the tumour microenvironment (TME) [3]. Melanoma CSCs are mainly characterized by upregulated levels of surface stem factors, including Nanog, Sox2, and Oct4, and their sphere formation capacity in vitro and in vivo [4, 5].

Although major efforts have been made in recent decades, useful therapeutic strategies targeting melanoma CSCs to address chemoresistance and radioresistance, which cause poor prognosis, remain challenging. Several candidate strategies have been proposed, but few have been applied clinically [6]. In treating glioblastoma stem cells, Pizzocri and colleagues employed drug-loaded liposomes and aimed to trigger an in situ immune response [7]. This method was found to be an effective strategy to deliver cytotoxic molecules to GSCs at the surgical tumour margins, which are the forefront of glioblastoma (GBM) recurrence, circumventing blood–brain barrier hurdles. Carrillo-Gálvez reported that glycoprotein A repetitions predominant (GARP) is a potential target on the surface of human osteo-, chondro-, and undifferentiated pleomorphic sarcomas. Targeting GARP in bone sarcomas could reduce tumour burden while simultaneously improving the efficacy of chemo- and radiotherapy [8]. All these results demonstrate that targeting CSCs is a potential and efficient strategy to overcome chemo- and radioresistance, which cause poor prognosis.

The last decades of research have led to the identification of a specific population of cancer cells endowed with the capability to self-renew and differentiate that are highly responsible for tumour growth and progression [9]. These cells, known as CSCs, possess intrinsic resistance to chemo- and radiotherapy, have high metastatic potential, and result in tumour relapse after treatment. Previously considered to be a small population, CSCs appear to be heterogeneous and sometimes numerous within specific types of cancer [10]. Due to their high plasticity, CSCs may experience phases of transition between stem-like and non-stem-like states. Furthermore, increasing evidence demonstrates that bulk tumour cells can acquire a stem cell-like phenotype in response to exogenous stimuli. This finding suggests that the process of cancer cell differentiation can be reversed and further contributes to cancer heterogeneity [9–11]. Altogether, considerable controversy remains as to how unequivocally define CSCs and to what extent distinct tumour types possess a hierarchical organization. Nevertheless, a growing body of evidence indicates that stem cell-associated molecular features, collectively known as stemness, are biologically important in cancer development and progression [9–11].

Natural herbs with a variety of biological and physiological effects have been widely employed in clinical practice for thousands of years worldwide. Traditional Chinese medicine is considered one of the most ancient medicines. Radix Astragali, Radix Ginseng, and Radix Codonopsis play an important role and exert significant therapeutic effects in melanoma therapy through many mechanisms and targets [12]. CHE is one of the main constituents of the genus *Chelidonium* L. [13], which can also be extracted from the herbs *Toddalia asiatica* (Linn) Lam [14] and *Macleaya cordata* (Willd.) R. Br [15]. CHEs have shown a variety of effects, including antitumour [16], antibacterial [14], anti-inflammatory [13], pesticidal, and antihepatic fibrosis effects [17], and certain protective effects against diabetic cardiomyopathy [18–20]. Due to its antitumour effects, CHE can inhibit the proliferation of lung cancer [21], liver cancer [22], and breast cancer cells [16] and induce apoptosis [19].

There is still a lack of research on the treatment of malignant melanoma with CHE [19]. It has been reported that CHE leads to ROS generation and accumulation, resulting in the inhibition of cell proliferation, reduction of colony formation, and induction of cell apoptosis [23]. In this study, we evaluated the effects of CHE on the stemness of melanoma CSCs by regulating ROS levels and mitochondrial function.

## 2. Material and Methods

### 2.1. Cell Culture and Enrichment of CSCs

Human melanoma A2058 and A375 cells were kept in culture dish (Corning Incorporated Life Sciences, Tewksbury, MA, USA), with the presence of 10% (*v*/*v*) fetal bovine serum (FBS, Gibco, Carlsbad, CA), 100 units/mL penicillin, and 100 *μ*g/mL streptomycin at 37°C under 100% humidity. Cells were passaged every 2-3 days.

For sphere formation, 2 × 10^5^ melanoma cells were seeded in 6-well plates (Corning Incorporated Life Science, NY, USA) and cultured in DMEM/F-12 (Gibco) without addition of FBS and supplemented 2% (*v*/*v*) B27, 10 ng/mL EGF, and 20 ng/mL bFGF. Medium was half-refreshed every 2-3 days.

### 2.2. Cell Viability

To evaluate cell viability, CCK-8 assay (Sigma Aldrich) was employed. Briefly, 5 × 10^3^ cells were seeded in 96-well plates and allowed to be cultured at 37°C under 100% humidity overnight. After 24, 48, 72, 96, or 120 h, 10 *μ*L of CCK-8 reagent was added to the medium and allowed for 2-hour incubation at 37°C. Then, the absorbance was read at 450 nm using the microplate reader (Bio-Rad, Milan, Italy).

### 2.3. Cellular and Mitochondrial ROS Quantification

To evaluate cellular ROS level, ROS-Glo H_2_O_2_ assay kit (Promega, Madison, WI, USA) was employed following the manufacturer's protocol. Detectable signal was analysed using Polarstar Optima plate reader (BMG LABTECH, Ortenberg, Germany). To analyse mitochondrial ROS, MitoSOX Red staining (Thermo Fisher) was employed following the manufacturer's protocol. Briefly, 5 *μ*mol/L of MitoSOX Red was added into medium for 10-minute incubation at 37°C and quantitatively measured using FACSCanto II.

### 2.4. Western Blot

20 *μ*g of total protein for each sample was fractionated by using 8-12% gradient SDS-PAGE, and fractionated bands were transferred onto a PVDF membrane, which was blocked by 5% (*w*/*v*) skim milk. Then, membrane was incubated in primary antibodies (1 : 1000 in 5% skim milk in TBST) at room temperature for 2 hrs. The antibodies employed were listed as follows: anti-Nanog antibody (ab109250, Abcam), anti-Sox2 antibody (ab92494, Abcam), anti-Oct4 antibody (ab109183, Abcam), and anti-*β*-actin antibody (Ab8226, Abcam). Then, the membrane was incubated with HRP-conjugated secondary antibody (1 : 10000, Ab270144, Abcam) for 2 hrs at room temperature followed by enhanced chemiluminescent detection (Millipore, Billerica, MA, U.S.A.).

### 2.5. Apoptosis

To evaluate cellular apoptosis rate, Annexin V-FITC/PI Apoptosis Detection Kit (Abcam, Cambridge, England) was used. 1 × 10^6^ cells were collected, washed with ice-cold PBS for three times, and resuspended in staining buffer with addition of Annexin V-FITC and PI according to the manufacturer's instructions. After 30 min incubation at room temperature avoiding light, cells were analysed by performing flow cytometry with 3 laser Navios flow cytometers (Beckman Coulter, Brea, CA, USA) in 30 min.

### 2.6. ATP Measurement

To quantitatively measure total ATP synthesis, ATP detection kit (LT07-221, ViaLight Plus kit, Lonza, Basel, Switzerland) was employed following the manufacturer's protocol. Briefly, 5 × 10^5^ cells were lysed for one vial analysis. Chemiluminescence was read in an FL ×800 microplate fluorescence reader (BioTek, Winooski, VT, USA).

### 2.7. Statistical Analysis

The experiments were performed at least five times for a reliable application of statistics. All samples used were included in the statistical analysis. Statistical analysis was performed by *T* test, one-way analysis of variance (ANOVA), and two-way ANOVA with GraphPad Prism 6 software, as specified in each figure legend. Statistical significances were accepted at *P* < 0.05. Values are presented as mean of independent experiments ± SD.

## 3. Results

### 3.1. Cancer Stem-Like Cells Derived from Melanoma Cells Are Sensitive to CHE

To obtain CSCs from A375 and A2058 cells, CSCs were enriched by culturing in serum-free medium and formed spheres were collected separately after 14 days (Figure 1(a)). In enriched A375 and A2058 CSCs, stem factors including Nanog, Oct4, and Sox2 were obviously increased compared with those in A375 and A2058 parental cells (Figure 1(b)). By performing cell viability assay, it was observed that enriched CSCs present slight decrease in A375 and A2058 CSCs compared with those in A375 and A2058 (Figure 1(c)).

To access CHE sensitivity to PCs or CSCs, 5-40 *μ*mol/L of CHE was cocultured with PCs or CSCs for 24 h and then cell viability was measured. It is observed that lower CHE concentration induced decrease in A375 and A2058 CSCs compared to those in A375 and A2058 PCs (Figures 2(a) and 2(b)). Notably, 30 *μ*mol/L of CHE slightly caused cellular apoptosis in both A375 and A2058 CSCs (Figure 2(c)), which indicated that low concentration of CHE (<30 *μ*mol/L) mainly induce cell cycle arrest but not apoptosis.

### 3.2. Relative Low Concentration of CHE Inhibits Stemness of Melanoma CSCs without Disturbing Cell Viability

To confirm the effects of CHE on stemness maintenance of CSCs derived from melanoma cells, we treated A375 and A2058 CSCs using 1-5 *μ*mol/L of CHE for 7 days. Morphologically, it is observed that CHE treatment decreased the formation of spheres and reduced the diameter of sphere observed (Figure 3(a)). To confirm whether the reduction of sphere formation is caused by cytotoxicity, CCK-8 assay was performed to evaluate the cell viability after 24 h treatment of different concentrations of CHE. Expectedly, 1-3 *μ*mol/L of CHE exerts no obvious effect on cell viability, while 4 and 5 *μ*mol/L of CHE decreased cell viability (Figure 3(b)). After a 7-day treatment, stem factors including Nanog, Oct4, and Sox2 were also decreased by 1-5 *μ*mol/L of CHE treatment (Figure 3(c)), indicating that 1-3 *μ*mol/L of CHE decreases stemness of melanoma CSCs without affecting cell viability.

### 3.3. CHE Inhibits Sphere Formation of Melanoma Cells

To evaluate whether CHE inhibits sphere formation of melanoma cells, we cultured melanoma cells in serum-free medium with the addition of 3 *μ*mol/L of CHE for 4-day incubation. Images were taken at the same position to observe the processes of sphere formation. As it is shown in Figures 4(a) and 4(b), the addition of CHE obviously inhibited sphere formation while melanoma cells were still stably attached to the bottom of wells, suggesting that CHE inhibits sphere formation, but does not exert cytotoxicity. CCK-8 assay further confirmed that CHE treatment slightly affected cell viability for 1-3 days (Figure 4(c)). It is expectedly observed that, after a 5-day incubation, stem factors including Nanog, Oct4, and Sox2 were not obviously upregulated when compared to the mock group (data not shown).

### 3.4. CHE Inhibits Intracellular and Mitochondrial ROS and Reduced ATP Synthesis

To examine the effects of CHE on cellular physiological processes, we examined the accumulation of cellular or mitochondrial ROS. We analysed cellular ROS and mitochondrial ROS, respectively. As it is shown in Figures 5(a) and 5(b), it is observed that the addition of 3 *μ*mol/L of CHE significantly increased both cellular and mitochondrial ROS levels. By adding NAC to 10 *μ*mol/L, the inhibitory effect of CHE on sphere formation was reversed (Figure 5(c)), suggesting that CHE-induced ROS accumulation is critical for its inhibitory role in stemness potentially via disturbing mitochondrial function.

Taken together, all results demonstrate that CHE affects stemness of melanoma CSCs potentially via inducing ROS accumulation and subsequently caused mitochondria-related energy disturbance.

## 4. Discussion

CHE exerts antitumour effects on various human tumour cell lines by inhibiting cell proliferation and inducing apoptosis [22, 24, 25]. However, its effects on CSCs are still largely unknown [25–27], which causes challenges and problems for its applications. In this study, we studied the in vitro effects of CHE on the stemness of melanoma CSCs and its potential mechanism of action. The addition of a relatively low concentration of CHE, which presents undetectable cytotoxicity and antitumour effects on melanoma cells, significantly reduced the stemness of melanoma CSCs, including A375 and A2058 CSCs. These results suggest that CHE regulates the maintenance of stemness in melanoma CSCs. Moreover, pretreatment with CHE inhibited sphere formation of melanoma cells. These findings further suggest that CHE not only inhibited stemness of melanoma CSCs but also inhibited sphere formation of CSCs.

In a previous report, chelerythrine hydrochloride (CHE) was shown to exert inhibitory effects on non-small-cell lung carcinoma- (NSCLC-) derived CSCs [28]. The dose–response pattern of CHE in three NSCLC cell lines showed a similar overall pattern of cytotoxicity and growth arrest over the entire concentration range, suggesting that CHE cytotoxicity exists globally. We examined the inhibitory effect of 5 to 40 *μ*mol/L CHE on cell viability in melanoma parental cells and related CSCs. Melanoma CSCs were more sensitive to the effects of CHE. A relatively low dose of CHE inhibited cell viability in both A375 and A2058 CSCs but not in their parental cells. Moreover, CHE failed to induce cell apoptosis, indicating that effects of CHE on cell viability were potentially due to blockage of cell cycle distribution. As a limitation of this study, we failed to analyse cell cycle distribution. We also observed that after treatment with chelerythrine at low concentrations, the spheres of melanoma cells disintegrated instead of undergoing cell death. There is one possible reason for this particular effect: the addition of CHE-differentiated melanoma cells and differentiated melanoma cancer cells results in tolerance to CHE.

The effects of CHE on CSCs were previously investigated. Zhu and colleagues reported that in NSCLC CSCs, CHE treatment downregulated the expression of Sox2, MYC, and *β*-catenin, which are critical stem factors. These results suggest that CHE may reduce CSC properties and induce apoptosis via the Wnt/*β*-catenin pathway [29]. In this study, we observed significant downregulation of Sox2 expression in melanoma CSCs and the expression of two other stem factors, Nanog and Oct4, which are critical for maintaining stemness. However, a decrease in *β*-catenin was not observed (data not shown), potentially due to the low endogenous level of *β*-catenin. To mimic the cytoplasmic accumulation and nuclear localization of *β*-catenin, we used GSK3i, a GSK3*β* inhibitor, to stimulate *β*-catenin levels. Surprisingly, the addition of GSK3i failed to induce *β*-catenin (data not shown), potentially because *β*-catenin is not critically regulated by GSK3*β*-*β*-catenin signalling.

Previous studies have demonstrated that ROS induce cell apoptosis by affecting mitochondrial function in cancer cells [30, 31], and CHE was reported to cause cell death by accumulating ROS in NSCLC cells [23]. In this study, consistent with previous findings, CHE treatment significantly induced cellular ROS and mitochondrial ROS accumulation in melanoma CSCs. Moreover, CHE treatment-induced inhibition of sphere formation was reversed by the addition of NAC, which is an ROS scavenger. These findings suggest that CHE-induced ROS are critical for the inhibitory role of CHE in the stemness of melanoma CSCs. Induction of ROS production from nicotinamide adenine dinucleotide phosphate oxidase, mitochondria, cyclooxygenase, etc., or a reduction in the scavenging capacity of ROS contributed to the intercellular accumulation of ROS [23, 32, 33]. Catalase is an enzyme that breaks down hydrogen peroxide in cells. This produces intercellular reactive oxygen species by selectively degrading the protein expression of catalase, leading to cell death [34]. Mitochondrial ROS, in most cases, enhance prosurvival autophagy and thus reduce cell apoptosis [35]. These findings indicate that the origin of ROS induced by CHE treatment may lead to different consequences in cancer therapy. In this study, intracellular ROS and mitochondrial ROS were all induced by CHE. This finding may explain why a relatively low dose of CHE inhibits cell proliferation and stemness but does not induce apoptosis. This issue should be clarified in the future. CHE critically affects mitochondria and malignancies in melanoma CSCs and is well recognized as a potent inhibitor of protein kinase C (PKC) for isoforms *α* and *β*. However, its effect on normal cells is still missing and worth investigating in further studies. CHE was also demonstrated to exert cell death-promoting effects in different manners, including apoptosis [36, 37] and necrotic-like cell death [38]. We only demonstrated the effects of CHE on apoptosis with or without NAC, although CHE treatment obviously induced necrotic-like cell death (Figure 2(c)). This also requires further investigation.

## 5. Conclusion

In this study, we observed that CHE probably inhibited melanoma CSC growth and stemness by inducing ROS accumulation and regulating mitochondrial function and energy production. CHE is considered an inhibitor of melanoma CSCs but also prevents melanoma cells from developing into melanoma CSCs. In further studies, we will identify the exact role of intracellular ROS and mitochondrial ROS in CSC fate to determine the optimal use of CHE in the clinical setting.

## Figures and Tables

**Figure 1:** Enrichment and characterization of CSCs derived from A375 and A2058 cells. (a) After being cultured in serum-free DMEM/F-12 medium, spheres formed were imaged and collected. (b) To identify stemness factors, Nanog, Oct4, and Sox2 were detected. ^∗^*P* < 0.05 vs. A375 PCs; ^#^*P* < 0.05 vs. A2058 PCs (*n* = 3). (c) The proliferating capacity of A375 or A2058 CSCs was detected by performing CCK-8 assay compared to which of PCs. ^∗^*P* < 0.05 vs. A2058 PC group (*n* = 3).

**Figure 2:** Melanoma CSCs were sensitive to CHE. (a) 5-40 *μ*mol/L of CHE was cocultured with A2058 and A375 CSCs or PCs for 24 h, and then, cell viability was measured by CCK-8 assay. (b) IC30 of CHE to cells were calculated. ^∗^*P* < 0.05 vs. PC group (*n* = 3). (c) After 30 or 40 *μ*mol/L CHE treatment for 24 h, cell apoptosis was measured by performing Annexin V-FITC/PI double staining followed by flow cytometry assay. ^∗^*P* < 0.05 vs. PC group (*n* = 3).

**Figure 3:** CHE inhibits stemness of melanoma CSCs without affecting cell viability. (a) 1-5 *μ*mol/L of CHE was cocultured with CSCs for 7 days, and morphological change of spheres was imaged. (b) CCK-8 assay was performed to detect the effect on cell viability after 24 h. ^∗^*P* < 0.05 vs. mock group (*n* = 3). (c) Western blot was performed to detect the stem factors, including Nanog, Oct, and Sox2. ^∗^*P* < 0.05 vs. mock group (*n* = 3).

**Figure 4:** CHE inhibits sphere formation of CSCs in serum-free medium. (a, b) After the addition of 3 *μ*mol/L of CHE for 24-96 h, cell morphology was imaged at the same position of each well. (c) Cell viability was measured after 24-96 h CHE treatment. ^∗^*P* < 0.05 vs. mock group (*n* = 3).

**Figure 5:** CHE increased ROS level and ATP function, which were reversed by NAC. After CHE treatment, with or without the presence of NAC, a ROS scavenger, (a) cellular ROS level was measured by ROS-Glo staining and (b) mitochondrial ROS was measured by MitoSOX Red staining. ^∗^*P* < 0.05 vs mock group; ^#^*P* < 0.05 vs CHE group (*n* = 3). (c) Sphere formation capacity was observed with the addition of NAC or CHE after 96 h incubation.

## Data Availability

The datasets generated and/or analysed during the current study are available from the corresponding author on reasonable request.
